# Clinical Application Value of Group-Sharing Nursing Management Based on Case Analysis

**DOI:** 10.1155/2022/1810573

**Published:** 2022-08-13

**Authors:** Jing Mei, Yifan Wu, Jie Hu, Min Li

**Affiliations:** ^1^Department of Nursing, Jiujiang First People's Hospital, Jiujiang, China; ^2^Thoracic Surgery, Jiujiang First People's Hospital, Jiujiang, China; ^3^Chest Pain Center, Jiujiang First People's Hospital, Jiujiang, China; ^4^Department of Nursing, Shanyang Traditional Chinese Medicine Hospital, Shangluo, China

## Abstract

The purpose of this study was to explore the clinical application value of group sharing nursing management based on a case analysis. The archive data of 90 nurses in 15 nursing units of our hospital were analyzed retrospectively. A total of 90 nurses from 15 nursing units in our hospital were retrospectively analyzed: the nurses before the implementation of the “case study-based group shared care management” program from January 2019 to January 2020 were set up as the control group, and the same nurses after the implementation of the program from January 2020 to January 2021 were set up as the study group. The nurses in the study group and the control group corresponded to 9759 and 8973 clinical inpatients, respectively. The overall incidence of medication-related, falling, tube-related, exam-related, and other types of adverse events was lower in the study group (0.52% vs. 1.29%) than those in the control group (*P* < 0.05); the overall nursing adverse event rating was lower in the study group than that in the control group (*P* < 0.05). Nurses in the study group scored higher than the control group on the following scales: Perceived Occupational Benefit Scale, General Self-Efficacy Scale, and Karlausk/Miller Satisfaction Scale (*P* < 0.05). The case study-based group-shared care management model can reduce the risk and harm of adverse events in hospitals and improve nurses' sense of professional benefit and self-efficacy.

## 1. Introduction

Adverse events in nursing care can be harmful and widespread, resulting not only in reduced clinical outcomes and increased financial costs of treatment, but also in patient disability or death [1, 2]. A large number of clinical studies [3, 4] have confirmed that case studies of nursing adverse events and sharing of experiences among nurses can effectively improve the efficiency of nursing management and reduce the risk of nursing adverse events, with the main methods including simulation exercises, nursing quality briefings, and summaries of monthly/quarterly nursing reports. However, the abovementioned sharing models generally suffer from inflexible sharing times and locations, cumbersome sharing processes, and long operational cycles. Clinical nurses are restricted by their management authority to access reported adverse events flexibly in order to optimize nursing measures, which makes it difficult for nurse leaders to make use of the information on the unit's abnormalities to strengthen nursing control measures in high-risk areas and limits the efficiency of nursing management. In our hospital, nursing management is carried out in groups of nurses and experience is shared within the nursing team based on the results of adverse event case analysis, which effectively improves the efficiency of the use of the information on the variation within the group as well as the management efficiency and achieves good results.

## 2. Materials and Methods

### 2.1. General Information

This was a historical controlled study, retrospectively analyzing the files of 90 nurses in 15 nursing units in our hospital from January 2019 to January 2021. The nurses before the implementation of “case study-based group shared care management” from January 2019 to January 2020 were set as the control group, and the same group of nurses after the implementation of “case study-based group-shared care management” was set up as the study group. The inclusion criteria were as follows: (i) the nurses were in nursing units with inpatient wards and inpatients, and had better nursing adverse event monitoring data; (ii) the nurses were all continuously employed in the same nursing unit from January 2019 to January 2021, and there were no adjustment changes in nursing quality control staff; (iii) the nurses all obtained the People's Republic of China nursing license. Nurses who took continuous leave of absence for ≥1 month during January 2019∼January 2021 were excluded. Nurses who have suffered medical errors in the course of their work were excluded. There was no statistically significant difference in the basic characteristics of the inpatients cared for during the study period between the two groups (*P* > 0.05), as shown in Table 1.

### 2.2. Methods

Nurses in the control group received routine nursing management; only the daily work content and completion of nurses were managed and assessed for quality evaluation every day. The nursing adverse events that occurred during nursing were truthfully reported in the adverse event reporting system of our hospital. Only the head nurse of each nursing unit had the permission to inquire about the adverse events and could only inquire about the relevant adverse events occurred in the nursing unit. The adverse events of other nurses and other nursing units could only be shared through the quarterly report on nursing quality issued by the nursing department.

The study group received group-shared nursing management based on case analysis: (1) nursing team establishment: we took the nursing unit as the basic unit, each nursing unit was an independent nursing team, each group of nurses was assigned 5∼10 people according to the actual situation, and the team leader was the head nurse. (2) Adverse event query authority definition: we flexibly opened up the nurses' adverse event query authority for each nursing unit, and the head nurse was able to query not only the nursing adverse events in her department, but also the occurrence of nursing adverse events in the whole hospital after getting approval by the nursing department. (3) Implementation of nursing target responsibility: firstly, the target responsibility of specialist nurses in the process of clinical patient care should be implemented and refined to every stage during the patient's hospitalization. We kept detailed records of the implementation of nurses' goals, which included specific goals such as psychological care goals, complication prevention goals, rehabilitation training goals, and nursing adverse event control goals. All of these nursing goals were implemented by the nurses according to the daily nursing care plan and the time of implementation is recorded, monitored, and evaluated by the nurses in the nursing team who were specifically responsible for assessment. (4) Adverse event reporting and case analysis: adverse events occurring in each nursing unit needed to be strictly classified and summarized for reporting, according to the type of adverse event, time of occurrence, nurse level, harm caused, and the way it was handled; during the study period, the head nurse applied for access to our hospital's adverse event platform at 9:00 a.m. every day on a fixed working day in the form of a work number, and the head nurse was granted access by the nursing department's backstage duty officer. After verification of the identity, the nurse manager was granted access to the platform to check the nursing adverse events that occurred within 48 hours in our hospital, and the nurse manager could choose to directly obtain the daily summary of the hospital-wide adverse events, which hid the private information of patients and nurses, and contained only the type of adverse events, time of occurrence, nurse level, harm caused, and handling methods. The head nurse will print out the daily summary and then call the whole group of nurses to conduct a case study, mainly focusing on the causes of adverse events, countermeasures, and prevention strategies to discuss and summarize the experience. (5) Group-sharing based on case analysis: during the daily case analysis of adverse events, the group discusses in the form of brainstorming, combining the results of the case analysis with the nurses' clinical nursing experience to summarize the prevention strategies and optimal solutions for the relevant nursing adverse events, and the nurse leader or experienced senior nurses will explain and share their experience in detail for the group members to improve their ability to respond to the situation. At the same time, the group should summarize the occurrence of adverse events in the whole hospital and the group in the corresponding period of time on a weekly, monthly, quarterly, semi-annual, and annual basis, and analyze and compare the adverse events in the whole hospital with those in the group to find out the problems and shortcomings of the group, and systematically collect and learn the operation methods and skills of adverse events through the literature research method every month. The team members share their learning experiences with each other to promote the overall improvement of the nurses' ability and skills in dealing with adverse events.

### 2.3. Observation Indicators

Incidence of adverse events: the incidence of adverse events during nursing care was counted for both groups. The main types of adverse events included drug-related, falls/bedding, tube-related, test/exam-related, and other types (pressure sores, wandering, burns, aspiration, etc.).

Severity of adverse events: according to the dangers and negative effects of adverse nursing events in the two groups, adverse events were divided into the following grades [5, 6]: (1) grade 1: adverse events had not been corrected before they occur, without causing factual effects; (2) grade 2: adverse nursing events had actually occurred, but had not caused physical and mental damage to patients; (3) grade 3: adverse nursing events had actually occurred, and this event has caused mild damage to the recoverability of patients' body functions; (4) grade 4: adverse nursing events had actually occurred, and this event had caused permanent loss of patients' body functions or led to patients' death. Among which, the adverse events of grade 1 were potential hazards, the adverse events of grade 2∼3 are minor adverse consequences, and the adverse events of grade 4 are serious adverse consequences.

Nurses' sense of occupational benefit and self-efficacy: at the end of the study in the two groups of nurses, the General Self-Efficacy Scale [7] (Cronbach's *α* coefficient 0.895) was used to assess nurses' self-efficacy, which had a total of 10 score items, each of which used a 4-level (1, 2, 3, and 4 points) score; the sum of the scores of each item divided by 10 was the total score, and the total score was 4 points, indicating that the self-efficacy was stronger; the Nurses' Sense of Occupational Benefit Scale [8] (Cronbach's *α* coefficient 0.921) was used to assess nurses' sense of occupational benefit, which included 5 subscales (Cronbach's *α* coefficient 0.873∼0.897) including positive sense of occupation (7 items), self-growth (6 items), nurse-patient relationship (7 items), team belonging (7 items), and approval of relatives and friends (6 items). Each item is scored using five levels (1, 2, 3, 4, and 5 points), with a total score of 33∼165 points, and the score is directly proportional to the nurses' sense of occupational benefit.

Nurse job satisfaction: at the end of the study in the two groups of nurses, the Karolsk/Miller Satisfaction Scale [9] (Cronbach's *α* coefficient 0.945) was used to evaluate nurse job satisfaction, which had a total of 31 items, and the nurse satisfaction of each item was scored using Likert grade 5, with a total score of 155, and a higher score indicated that the nurses were more satisfied with the work.

### 2.4. Statistical Analysis

Statistical Product and Service Solutions (SPSS) 23.0 (IBM, Armonk, NY, USA) was applied for statistical analysis. The independent sample *t*-test was used for comparison between groups for measurement data obeying normal distribution, and the independent sample *t*-test was used for comparison within groups, all data are expressed as ($\bar{x}\pm s$). Count data were tested by *χ*^2^ and expressed as rate (%), *P* < 0.05 indicates statistical difference.

## 3. Results

### 3.1. The Incidence of Adverse Events between the Two Groups

The overall incidence of drug-related, fall/fall, tubing-related, test/examination-related, and other types of adverse events in the study group (0.52% vs. 1.29%) was lower than that in the control group (*χ*^2^ = 31.360, *P* < 0.05) (Table 2).

### 3.2. Adverse Event Grades between the Two Groups

The grade of adverse nursing events in study group was generally lower than that in the control group, and the difference between the two groups had a statistical significance (*Z* = 9.331, *P* < 0.05) (Table 3).

### 3.3. Occupational Benefit between Two Groups of Nurses

Nurses in the study group had higher positive sense of occupation (*t* = 3.074), their own growth (*t* = 3.441), nurse-patient relationship (*t* = 2.873), team affiliation (*t* = 2.528), identification of relatives and friends (*t* = 3.055), and total score (*t* = 6.524) than those in the control group (Fig. *P* < 0.05) (Table 4).

### 3.4. Self-Efficacy and Job Satisfaction between Two Groups of Nurses

The scores of the General Self-Efficacy Scale (*t* = 7.948) and Karsk/Miller satisfaction scale (*t* = 3.512) of nurses in the study group were higher than those in the control group (*P* < 0.05) (Table 5).

## 4. Discussion

Adverse events in nursing care are clinically defined as unanticipated events during care that may cause the patient to receive physical or psychological harm, including unnatural accidents such as a patient falling out of bed, wandering, falling, aspiration, and dislodging a blood or fluid line during hospitalization [10, 11]. A relevant report by the World Health Organization (WHO) [12] showed that the chance of accidental injury to patients treated in developed countries was 10%, and about 40% of these injured patients were caused by nursing accidents. The focus of hospital nursing management has always been on how to improve the overall treatment effect and medical experience while ensuring the physical and psychological comfort of patients. With the continuous improvement of clinical requirements for the quality of medical services and nursing staff, as the group with the most frequent clinical contact with patients, the improvement of their professional level, core skill mastery, and adaptability is of great significance for medical service centers to improve the quality of medical services [13]. For a long time, in order to reduce the incidence of nursing adverse events, and improve the professional literacy of nursing staff and the quality of hospital services, hospitals have been committed to finding an adverse event sharing management model with strong operability, advanced concept, and good application effect, while the information sharing of simulation drills, nursing quality briefing, and other methods has a certain lag, and there are many restrictions on the rights of nurses, which is not conducive to the sharing and transmission of nurses' adverse event processing experience [14, 15].

The results of this study showed that the total incidence rate of drug-related, fall/fall, tube-related, test/examination related, and other types of adverse events in study group (0.52% vs. 1.29%) was lower than that in control group, and the nursing adverse event grade in study group was generally lower than that in control group, indicating that group-shared nursing management based on case analysis could reduce the overall risk of nursing adverse events and the degree of harm of adverse events. The results also showed that the scores of occupational benefits, self-efficacy, and the job satisfaction scale of nurses in the study group were higher than those in the control group, indicating that group-shared nursing management based on case analysis could also improve nurses' work enthusiasm and efficacy. Analyze the reason: because the group sharing nursing management model based on case analysis is improved on the basis of simulation drill, nursing quality briefing, and other methods, by appropriately increasing the adverse event inquiry authority of nurses, group cooperative case analysis, and the experience sharing method to improve the efficiency of abnormal information transmission among nurses not only help nurses grasp the occurrence of adverse events in this nursing unit and even the whole hospital more timely and accurately, but also nurses can learn lessons from the corresponding adverse event cases and combine them with case analysis to find out and fill the gaps in the nurses' own nursing theory and skill knowledge level, and improve the prevention and control the level of adverse events and accident handling ability. On the other hand, under the group sharing nursing management model based on case analysis, there are many interaction contents between individual nurses and groups, and the sense of nurse participation is significant, which also greatly improves the sense of occupational benefit, self-efficacy, and work satisfaction of nurses, and can promote the construction of the hospital talent team and the improvement of medical service quality. The sample of this retrospective study is small, weakening the evidence of the findings, thus should be further verified by future studies with a large sample.

## 5. Conclusion

In summary, the clinical application effect of group-shared nursing management mode based on case analysis is good and exact, which can not only improve the prevention and control level of adverse events in nurses, and reduce the risk and harm of adverse events in hospitals, but also improve the occupational benefit and self-efficacy of nurses, with a clinical promotion value.

## Figures and Tables

**Table 1:** Comparison of baseline data of nursing patients between the two groups.

Group	*N*	Age	Gender [*n*, (%)]		Reason for hospitalization [*n*, (%)]		
			Male	Female	Surgery	Critical illness	Emergency
Study group	9759	49.9 ± 4.33	5172 (53.00)	4587 (47.00)	4299 (44.05)	2205 (22.60)	3255 (33.35)
Control group	8973	50.05 ± 4.12	4678 (52.13)	4295 (47.87)	3989 (44.46)	2045 (22.79)	2939 (32.75)
*t*/*χ*^2^		1.473	1.397		0.761		
*P*		0.141	0.237		1.684		

**Table 2:** Comparison of incidence rate of adverse events between the two groups [*n*, (%)].

Group	*N*	Drug-related	Fall/bed drop	Tubing related	Inspection/inspection related	Other types	Total
Study group	9759	10 (0.10)	19 (0.19)	6 (0.06)	4 (0.04)	12 (0.12)	51 (0.52)
Control group	8973	22 (0.25)	45 (0.50)	18 (0.20)	10 (0.11)	21 (0.23)	116 (1.29)
*χ * ^2^							31.360
*P*							<0.001

**Table 3:** Comparison of adverse event grades between the two groups [*n*, (%)].

Group	*N*	Level 1	Grade 2	Grade 3	Grade 4
Study group	51	42 (82.35)	5 (9.80)	4 (7.84)	0
Control group	116	68 (58.62)	32 (27.59)	15 (12.93)	1 (0.86)
*Z*					9.331
*P*					0.025

**Table 4:** Comparison of improvement in nurses' sense of occupational benefit (i.e., $\bar{x}\pm s$, minutes).

Group	*N*	Positive sense of occupation	Self-growth	Nurse-patient relationship	Team assignments	Affirmative	Total score
Study group	90	20.15 ± 3.26	18.78 ± 4.15	20.30 ± 3.75	19.58 ± 4.87	18.69 ± 4.13	78.56 ± 7.33
Control group	90	25.02 ± 4.12	24.59 ± 3.76	25.12 ± 4.11	24.65 ± 4.53	23.73 ± 3.59	97.38 ± 6.15
*t*/*χ*^2^		3.074	3.441	2.873	2.528	3.055	6.524
*P*		0.006	0.003	0.009	0.020	0.006	<0.001

**Table 5:** Comparison between nurses' self-efficacy and job satisfaction (Fig. $\bar{x}\pm s$, minutes).

Group	*N*	General Self-Efficacy Scale	Kallusk/Miller satisfaction scale
Study group	90	2.05 ± 0.37	117.43 ± 19.53
Control group	90	3.56 ± 0.51	138.95 ± 5.62
*t*/*χ*^2^		7.948	3.512
*P*		<0.001	0.002

## Data Availability

The datasets used and analyzed during the current study are available from the corresponding author upon reasonable request.
